# Suicide Ideation among Outpatients with Alcohol Use Disorder

**DOI:** 10.1155/2022/4138629

**Published:** 2022-02-12

**Authors:** Wen-Yu Hsu, Ting-Gang Chang, Cheng-Chen Chang, Nan-Ying Chiu, Chieh-Hsin Lin, Hsien-Yuan Lane

**Affiliations:** ^1^Institute of Clinical Medical Science, China Medical University, Taichung 40402, Taiwan; ^2^Department of Psychiatry, Changhua Christian Hospital, Changhua 50006, Taiwan; ^3^School of Medicine, Chung Shan Medical University, Taichung 40201, Taiwan; ^4^Department of Psychiatry, Taichung Veteran General Hospital, Taichung 40705, Taiwanvghtc.gov.tw; ^5^Graduate Institute of Biomedical Sciences, China Medical University, Taichung 40402, Taiwan; ^6^Psychiatry, Kaohsiung Chang Gung Memorial Hospital, Kaohsiung 83301, Taiwan; ^7^School of Medicine, Chang Gung University, Taoyuan 33302, Taiwan; ^8^Department of Psychiatry & Brain Disease Research Center, China Medical University and Hospital, Taichung 40402, Taiwan; ^9^Department of Psychology, College of Medical and Health Sciences, Asia University, Taichung 41354, Taiwan

## Abstract

**Introduction:**

Individuals with substance use disorders, particularly those with alcohol use disorder (AUD), have a high risk of suicide. Therefore, identifying risk factors for suicide in these individuals is crucial.

**Methods:**

This retrospective study reviewed the medical records of individuals with AUD who participated in an alcohol treatment program in central Taiwan during 2019–2020. We collected data using the Cut down, Annoyed, Guilty, and Eye-opener questionnaire, Alcohol Use Disorders Identification Test (AUDIT), Brief Michigan Alcoholism Screening Test (MAST), Beck Depression Inventory (BDI), Beck Anxiety Inventory (BAI), and a suicidal ideation question. Furthermore, we collected information on several related variables, namely, sex, age, marital status, years in school, employment status, family history of alcohol problems, age at first exposure to alcohol, duration of alcohol use, history of alcohol cessation, history of domestic violence, and history of drunk driving. In total, 136 individuals were recruited to participate in this study.

**Results:**

The suicidal ideation group had significantly younger participants, a higher proportion of women, a higher proportion of participants with a history of domestic violence, a greater severity of alcohol addiction (based on both AUDIT and MAST scores), higher depression scores, higher anxiety scores, less social support, a lower quality of life (World Health Organization Quality of Life (WHOQOL)), and poorer sleep quality (Pittsburgh Sleep Quality Index, PSQI) compared with the nonsuicidal ideation group. The suicidal ideation score was correlated with the AUDIT score after age, and BDI, BAI, WHOQOL, and PSQI scores were controlled for (*P* = 0.034).

**Conclusion:**

Individuals with higher AUDIT scores visiting a clinic for alcohol treatment might have a higher risk of suicidal ideation. Therefore, clinicians should pay close attention to the suicidal ideation problem in this population. Furthermore, appropriate medication or management programs for suicide prevention should be considered.

## 1. Introduction

The prevalence of alcohol use disorder (AUD) and binge drinking has been increasing worldwide [1, 2]. AUD is among the most disabling mental disorders and is associated with some outcomes such as mortality and loss of disability-adjusted life years (DALY) [3, 4]. AUD is related to several physical comorbidities and complications such as alcoholic hepatitis, gastritis, pancreatitis, Wernicke–Korsakoff syndrome, cancer, diabetes, and accident injury [5, 6]. In addition, AUD is associated with mental disorders such as bipolar disorder, major depressive disorder, generalized anxiety disorder, personality disorder, phobia, and schizophrenia [7, 8]. Suicidal ideation often accompanies these disorders. Moreover, suicidal ideation and suicide attempt are not rare in patients with AUD. The risk of suicide is relatively high in patients with substance use disorders, particularly in those with AUD [9, 10]. According to a review of psychological autopsy studies, 19%–63% of individuals who completed suicide had substance use disorders [9]. Substance-related disorders were suggested to be strongly associated with an increased risk of completed suicide [11]. A meta-analysis demonstrated significant associations of AUD with suicidal ideation (odds ratio (OR) = 1.86; 95%confidence interval (CI) = 1.38, 2.35), suicide attempt (OR = 3.13; 95%CI = 2.45, 3.81), and completed suicide (OR = 2.59; 95%CI = 1.95, 3.23; risk ratio = 1.74; 95%CI = 1.26, 2.21) [12]. Furthermore, a meta-analysis of postmortem case–control studies revealed that individuals with AUD had a higher OR (3.68) than did those without AUD (95%CI = 1.99, 6.82) [13]. Furthermore, a longitudinal cohort study in Denmark reported that individuals with AUD had a significantly higher risk of completed suicide (crude hazard ratio [HR] = 7.98; 95%CI = 5.27, 12.07) than did those without AUD [14]; however, after adjustment for all psychiatric disorders, the crude HR (representing the risk of completed suicide) decreased to 3.23 (95%CI = 1.96, 5.33) [14]. In the aforementioned study in Denmark, a subgroup analysis involving individuals without psychiatric disorders indicated that the risk of completed suicide was 9.69 (95%CI = 4.88, 19.25) among individuals with AUD [14]. AUD is a major contributor to suicide rates at the population level [15]. Therefore, identifying the risk of suicide in patients with substance use disorders, particularly in those with AUD, is crucial for clinical physicians. Understanding the prevalence and severity of suicidal ideation in patients with AUD in outpatient settings is crucial for the prevention of suicide. However, studies on these topics in the Asian population are limited. To fill this research gap, we conducted this retrospective study to investigate the prevalence and severity of suicidal ideation in patients with AUD in an outpatient alcohol treatment program. Furthermore, we investigated the association between suicidal ideation and the severity of AUD.

## 2. Methods

### 2.1. Study Population

In this retrospective study, we collected relevant data from the medical records of patients who participated in an outpatient alcohol treatment program at Changhua Christian Hospital between January 2019 and December 2020. On the basis of the legal definition of adulthood in Taiwan, we excluded patients aged <20 years. The study protocol was approved by the Institutional Review Board of Changhua Christian Hospital. No commercial funding was acquired for this study. A total of 136 Taiwanese individuals were recruited for this study, and relevant data were analyzed, as described in the following section.

### 2.2. Alcohol-Related Data

We used the four-item Chinese version of the Cut down, Annoyed, Guilty, and Eye-opener questionnaire (C-CAGE)—a brief and effective questionnaire for screening alcohol problems—as the first screening tool [16, 17]. Furthermore, we used the Chinese version of the Alcohol Use Disorders Identification Test (C-AUDIT) and the Brief Michigan Alcoholism Screening Test (MAST) to identify patients with recent AUD and determine the severity of AUD [18–20]. AUD was diagnosed through an interview by psychiatrists on the basis of the *Diagnostic and Statistical Manual of Mental Disorders, Fifth Edition*, criteria. Furthermore, we collected the following variables related to alcohol use: sex, age, marital status, years in school, employment status, family history of alcohol problems, age at first exposure to alcohol, duration of alcohol use, history of alcohol cessation, history of domestic violence, and history of drunk driving. We also collected laboratory data, including gamma glutamyl transpeptidase, aspartate aminotransferase, aspartate aminotransferase, alanine aminotransferase, triglyceride, and total cholesterol levels.

### 2.3. Suicide Assessment and Related Scales

At the first clinic visit, the participants were asked if they had had any suicidal ideation in the previous month. We used the Chinese version of the Beck Depression Inventory (C-BDI) to determine the severity of depression and suicidal ideation [21]. A total BDI score of >13 indicates a depressive disorder. In this study, participants who provided an affirmative response to the suicidal ideation question or endorsed any suicidal thoughts on the suicide item of the C-BDI were assigned to the suicidal ideation group; those who did not provide an affirmative response to the suicidal ideation question or did not endorse any suicidal thoughts on the suicide item of the C-BDI were assigned to the nonsuicidal ideation group. Furthermore, we assessed anxiety status by using the Chinese version of Beck's Anxiety Inventory (C-BAI). A total BAI score of >7 indicates anxiety disorder. We assessed social support by using a self-report questionnaire. Specifically, two dimensions of social support were assessed, namely, perceived versus received social support and social support received under routine versus crisis status, resulting in four subscales: (i) perceived crisis support, (ii) perceived routine support, (iii) received crisis support, and (iv) received routine support [22]. We also evaluated quality of life by using the Taiwanese version of the World Health Organization Quality of Life (WHOQOL) questionnaire [23]. We applied the Chinese version of the Pittsburgh Sleep Quality Index (C-PSQI)—a self-administered questionnaire for evaluating subjective sleep quality during the previous month—to assess sleep quality [24]. In addition, we assessed the stress and mental health status of the family members accompanying the participants (hereafter referred to as main caregivers). We used the Chinese version of the Kingston Caregiver Stress Scale (C-KCSS) for stress assessment, and we applied the 12-item Chinese Health Questionnaire (CHQ-12)—a screening instrument for anxiety, depression, insomnia, fatigue, social functioning, and family relationships—to assess the mental health status of the main caregivers [25, 26].

### 2.4. Statistical Analysis

Demographic data are presented as mean and standard deviation values for continuous variables and as percentages for discrete variables. The prevalence of sex, family history of alcohol problems, employment status, marital status, depressive disorder, and anxiety disorder was calculated for each group, and the corresponding 95% Clopper–Pearson confidence intervals were estimated. For the univariate analysis of categorical variables, the chi-square and Fisher's exact tests were used. Furthermore, continuous variables were analyzed using Student's *t*-test and one-way analysis of variance with post hoc adjustments as required. Associations between suicidal ideation scores and continuous variables were calculated using Pearson's correlation analysis. Statistical analyses were performed using SPSS PC 22.0 software (SPSS Inc., Chicago, IL, USA).

## 3. Results

We recruited a total of 136 patients with AUD to participate in this study. Of the participants, 15 (11.03%) were women. Regarding employment status, 99 (72.79%) and 37 (27.21%) participants were employed and unemployed, respectively. Moreover, concerning age at first alcohol exposure, 38 (27.94%), 63 (46.32%), 27 (19.85%), and 8 (5.88%) participants began drinking alcohol in their teens (between 13 and 20 years), in their 20s (between 21 and 30 years), in their 30s (between 31 and 40 years), and after the age of 40 years, respectively. Regarding alcohol use duration, 58 (42.65%), 28 (20.59%), 18 (13.24%), 19 (13.97%), and 12 (8.82%) participants had been drinking alcohol for >20, 16–20, 11–15, 5–10, and<5 years, respectively. Furthermore, 32 (23.53%) participants reported having suicidal ideation. Regarding marital status, 80 (58.82%), 31 (22.79%), 21 (15.44%), and 2 (1.47%) participants were married, single, divorced, and separated, respectively. We also observed that 53 (38.97%) participants visited our clinic for the first time to quit alcohol. In addition, 20 (14.71%) participants had a history of domestic violence, and 76 (55.88%) participants had a history of drunk driving. The mean age of the study participants was 45.89 ± 10.79 years. The mean C-CAGE, MAST, and C-AUDIT scores for the study participants were 2.82 ± 0.96, 4.43 ± 1.76, and 25.69 ± 7.10, respectively. Moreover, the mean C-BDI and C-BAI scores were 18.21 ± 12.48 and 13.18 ± 12.00, respectively. The mean score of the suicidal ideation item of the C-BDI was 0.54 ± 0.85. The mean scores of social support and quality of life (WHOQOL) were 110.11 ± 17.66 and 86.55 ± 16.20, respectively. Additionally, the mean score of the C-PSQI was 12.24 ± 7.01. Finally, the mean scores of the C-KCSS and CHQ-12 for the main caregivers were 24.13 ± 10.05 and 26.77 ± 6.52, respectively.

We observed that the suicidal ideation group had a significantly younger age, a higher proportion of women, a higher proportion of participants with a history of domestic violence, greater severity of alcohol addiction (C-AUDIT and MAST), greater depression (C-BDI), more severe anxiety (C-BAI), lower social support, lower quality of life (WHOQOL), and poorer sleep quality (C-PSQI) than did the nonsuicidal ideation group.  Table 1 presents a summary of the aforementioned analysis results.

Female participants had significantly higher suicidal ideation scores than did male participants. Participants with a history of domestic violence, depressive disorder, or anxiety disorder had significantly higher suicidal ideation scores than did those without a history of domestic violence, depressive disorder, or anxiety disorder, respectively.  Table 2 presents the suicide severity analysis results for different categorical variables.

Our Pearson correlation analysis results revealed that the suicidal ideation score was associated with age (*P* < 0.001) and with MAST (*P* = 0.022), C-BDI (*P* < 0.001), C-BAI (*P* < 0.001), WHOQOL (*P* < 0.001), and C-PSQI (*P* = 0.001) scores. However, after controlling for age and C-BDI, C-BAI, WHOQOL, and C-PSQI scores, we observed that the suicidal ideation score was correlated with the C-AUDIT score (*P* = 0.034) but not with the C-CAGE (*P* = 0.151) or MAST (*P* = 0.729) scores.

## 4. Discussion

In this study, we assessed participants with AUD at their first clinic visit for the purpose of alcohol cessation and observed that 23.53% of them had suicidal ideation. Participants who were young, were women, had a history of domestic violence, had depression, had anxiety, had poor social support, had poor quality of life, had poor sleep quality, and had severe alcohol addiction constituted a high proportion of the participants with AUD who had suicidal ideation. Furthermore, the suicidal ideation score was correlated with age, alcohol severity, depression severity, anxiety severity, quality of life, and sleep quality. By contrast, the suicidal ideation score was not correlated with alcohol severity after age, depression severity, anxiety severity, quality of life, and sleep quality were controlled for.

A previous meta-analysis revealed that AUD was significantly associated with an increased risk of suicidal ideation, suicide attempt, and completed suicide [12]. However, studies on the prevalence of suicidal ideation and factors associated with suicidal ideation among outpatients with AUD are limited. Connor and colleagues found that suicidal ideation was common among women (15.5%) and men (9.9%) initiating treatment [27]. In our study, we observed that 23.53% of the participants with AUD (46.7% of whom were women and 20.7% were men) who were assessed at the first visit to our outpatient alcohol treatment program had suicidal ideation in the past month. The mean score of the suicide item of the C-BDI was 0.54 ± 0.85. These results demonstrate a high prevalence and severity of suicidal ideation in this population. Therefore, suicidal ideation is a critical problem in the clinical treatment of AUD. From a clinical perspective, identifying individuals at risk of suicidal ideation is necessary for the implementation of preventive interventions.

Through further analysis, we observed that participants with AUD who had suicidal ideation were younger than those without suicidal ideation. We also observed a significant association between age and depressive disorder. This might explain why the suicidal ideation group had a higher proportion of younger participants than did the other group. Our results reveal that the suicidal ideation group had a higher proportion of female participants. This finding is consistent with that of Connor et al., who reported that suicidal ideation was more common in women (15.5%) than in men (9.9%) [27]. Our finding is also consistent with that of Agrawal et al., who indicated that women with AUD had a 3.1 odds of reporting a lifetime history of suicidal ideation, which was higher than that observed for men with AUD [28]. In this study, the prevalence of depression and anxiety was also determined to be higher in women than in men in the AUD population. Women may consume alcohol in an attempt to coping with depression or anxiety. Furthermore, a history of domestic violence was associated with suicidal ideation in our study. Several studies have also reported domestic violence or criminal offense to be a risk factor for suicidal ideation [29, 30].

In our study, we found that the suicidal ideation group had higher AUD severity compared with the nonsuicidal ideation group. The suicidal ideation score was correlated with the C-AUDIT score after age, and C-BDI, C-BAI, WHOQOL, and C-PSQI scores were controlled for. Individuals with higher C-AUDIT scores might be at a higher risk of suicidal ideation. Conner et al. revealed that the quantity of alcohol consumed and frequency of alcohol consumption were associated with suicidal ideation in individuals initiating treatment for AUD [31]. They also found depression to be a partial or complete mediator of the association between alcohol drinking and suicidal ideation [32]. Accordingly, the results of our study are consistent with those of previous studies.

According to our results, suicidal ideation is related to the severity of alcohol addiction. Nevertheless, the cause and effect of both are unknown. Suicidal ideation might lead to increased alcohol consumption and addiction severity. Long-term alcohol use might increase impulsivity, emotion dysregulation, or cognitive deficits. These might increase the risk of suicidal ideation.

Our study has several limitations, which provide directions for future research. First, our study involved a retrospective design. Additional prospective studies on suicidal ideation monitoring could be helpful to provide stronger evidence. Second, our study sample was small. Hence, future research with a larger sample size might be necessary. Third, we used a self-report questionnaire for suicidal ideation assessment. A comprehensive interview for assessing suicidal ideation might provide more precise results regarding suicidal ideation.

Identifying patients with a high risk of suicide is the first step toward suicide prevention. Further comprehensive assessment of suicidal ideation is still necessary. Suicide prevention programs, including psychological interventions, behavioral interventions, supportive system enhancement, medication treatment, or professional referrals, should be considered for such patients.

In this study, we demonstrated that the prevalence and severity of suicidal ideation were high in Asian patients with AUD. The female sex, a young age, a history of domestic violence, the severity of alcohol addiction, depression, anxiety, poor social support, poor quality of life, and poor sleep quality could be associated with suicidal ideation in this population. Patients with higher C-AUDIT scores might have a higher risk of suicidal ideation; therefore, clinicians should focus on suicide management for these patients. Furthermore, the cause and effect of suicidal ideation severity and alcohol addiction severity, the change in suicidal ideation severity during alcohol treatment, and the association between alcohol addiction severity and suicidal ideation severity after alcohol treatment warrant further research.

## Figures and Tables

**Table 1:** Difference between patients in nonsuicide ideation group and patients in suicide ideation group in age, gender, employment, alcohol family history, first alcohol drinking age, alcohol use duration, alcohol quit history, domestic violence history, drunk driving history, gamma glutamyl transpeptidase, aspartate aminotransferase, alanine aminotransferase, triglyceride, total cholesterol, C-CAGE, C-AUDIT, MAST, C-BDI, C-BAI, social support score, WHOQOL, C-PSQI, C-KCSS, and CHQ-12.

	Nonsuicide ideation group *N* = 82 (mean ± SD)	Suicide ideation group *N* = 54 (mean ± SD)	*P*
Age (years)	48.07 ± 11.21	42.57 ± 9.26	0.002^∗^
Male gender (%)	96.34	77.78	0.001^#^
Empolyed (%)	73.17	72.22	1.000
Family alcohol problems (%)	24.39	31.48	0.432
First alcohol drinking age			0.564
Teenager (%)	28.05	27.78	
20~29 years old (%)	45.12	48.15	
30~39 years old (%)	18.29	22.22	
40 ~ years old (%)	8.54	1.85	
Duration of alcohol use			0.154
More than 20 years (%)	46.34	37.04	
16-20 years (%)	19.51	22.22	
11-15 years (%)	7.32	22.22	
5-10 years (%)	14.63	12.96	
Less than 5 years (%)	10.98	5.56	
Alcohol quit history (%)	58.54	64.81	0.479
Domestic violence history (%)	7.32	25.93	0.005^#^
Drunk driving history (%)	53.66	59.26	0.598
Gamma glutamyl transpeptidase (IU/L)	292.45 ± 442.03	307.06 ± 473.09	0.860
Aspartate aminotransferase (IU/L)	85.26 ± 114.47	77.88 ± 86.56	0.702
Alanine aminotransferase (IU/L)	62.39 ± 84.26	45.94 ± 32.41	0.129
Triglyceride (mg/dl)	249.99 ± 445.71	243.78 ± 355.84	0.936
Total cholesterol (mg/dl)	176.95 ± 47.16	180.92 ± 57.28	0.673
C-CAGE	2.70 ± 0.99	3.00 ± 0.90	0.082
C-AUDIT	24.50 ± 6.82	27.50 ± 7.20	0.015^∗^
MAST	4.10 ± 1.74	4.94 ± 1.68	0.006^∗^
C-BDI	11.69 ± 8.88	27.29 ± 11.04	<0.001^∗∗^
C-BAI	8.62 ± 7.06	19.71 ± 14.46	<0.001^∗∗^
Social support score	114.13 ± 12.83	104.45 ± 21.71	0.006^∗^
WHOQOL	93.65 ± 13.74	76.53 ± 14.04	<0.001^∗∗^
C-PSQI	10.38 ± 6.15	14.98 ± 7.36	<0.001^∗∗^
C-KCSS	23.57 ± 10.66	25.12 ± 9.00	0.541
CHQ-12	26.75 ± 6.85	26.80 ± 6.02	0.976

C-CAGE: Chinese version CAGE questionnaire; C-AUDIT: Chinese version Alcohol Use Disorders Identification Test; MAST: Brief Michigan Alcoholism Screening Test; C-BDI: Chinese version of Beck Depression Inventory; C-BAI: Chinese version of Beck Anxiety Inventory, Social support score; WHOQOL: Taiwan version World Health Organization Quality of Life; C-PSQI: Chinese version of Pittsburgh Sleep Quality Index; C-KCSS: Chinese version of Kingston Caregiver Stress Scale; CHQ-12: 12-item Chinese Health Questionnaire. Student's *t*-test and one-way analysis of variance ^∗^*P* < 0.05, ^∗∗^*P* < 0.001. Chi-squared test ^#^*P* < 0.05, ^##^*P* < 0.001.

**Table 2:** Suicide severity analyses in different categorical variables.

	Suicide idea severity score (mean ± SD)	*n*	*P* values
Gender			0.002^∗^
Male	0.46 ± 0.79	113	
Female	1.21 ± 1.05	14	
Education			0.762
Elementary school	0.33 ± 0.49	12	
Junior high school	0.67 ± 0.96	39	
Senior high school	0.49 ± 0.83	47	
2 years college	0.58 ± 0.90	12	
4 years college	0.60 ± 0.91	15	
Others	0.00 ± 0.00	2	
First alcohol drinking age			0.521
Teenager	0.58 ± 0.89	38	
20~29 years old	0.60 ± 0.88	58	
30~39 years old	0.50 ± 0.83	24	
40 ~ years old	0.00 ± 0.00	7	
Duration of alcohol use			0.267
More than 20 years	0.47 ± 0.81	55	
16-20 years	0.56 ± 0.89	27	
11-15 years	0.94 ± 0.85	16	
5-10 years	0.65 ± 1.00	17	
Less than 5 years	0.18 ± 0.60	11	
Job			0.902
Employed	0.54 ± 0.82	93	
Unemployed	0.56 ± 0.96	34	
Family history			0.814
Yes	0.51 ± 0.78	35	
No	0.55 ± 0.88	92	
Domestic violence history			0.001^∗^
Yes	1.10 ± 1.02	20	
No	0.44 ± 0.78	107	
Drunk driving history			0.218
Yes	0.63 ± 0.91	72	
No	0.44 ± 0.76	55	
Alcohol quit history			0.646
Yes	0.57 ± 0.87	77	
No	0.50 ± 0.84	50	
Depressive disorder			<0.001^∗∗^
Yes	0.93 ± 0.99	67	
No	0.13 ± 0.34	55	
Anxiety disorder			<0.001^∗∗^
Yes	0.76 ± 0.98	76	
No	0.22 ± 0.47	46	

Student's *t*-test ^∗^*P* < 0.05, ^∗∗^*P* < 0.001.

## Data Availability

The data that support the findings of this study are available on request from the corresponding author. The data are not publicly available due to privacy or ethical restrictions.
